# The Influences of Canopy Species and Topographic Variables on Understory Species Diversity and Composition in Coniferous Forests

**DOI:** 10.1155/2014/252489

**Published:** 2014-07-06

**Authors:** Hong Huo, Qi Feng, Yong-hong Su

**Affiliations:** ^1^Key Laboratory of Ecohydrology of Inland River Basin, Cold and Arid Regions Environmental and Engineering Research Institute, Chinese Academy of Sciences, Lanzhou 730000, China; ^2^University of Chinese Academy of Sciences, Beijing 100049, China

## Abstract

Understanding the factors that influence the distribution of understory vegetation is important for biological conservation and forest management. We compared understory species composition by multi-response permutation procedure and indicator species analysis between plots dominated by Qinghai spruce (*Picea crassifolia *Kom.) and Qilian juniper (*Sabina przewalskii* Kom.) in coniferous forests of the Qilian Mountains, northwestern China. Understory species composition differed markedly between the forest types. Many heliophilous species were significantly associated with juniper forest, while only one species was indicative of spruce forest. Using constrained ordination and the variation partitioning model, we quantitatively assessed the relative effects of two sets of explanatory variables on understory species composition. The results showed that topographic variables had higher explanatory power than did site conditions for understory plant distributions. However, a large amount of the variation in understory species composition remained unexplained. Forward selection revealed that understory species distributions were primarily affected by elevation and aspect. Juniper forest had higher species richness and *α*-diversity and lower *β*-diversity in the herb layer of the understory plant community than spruce forest, suggesting that the former may be more important in maintaining understory biodiversity and community stability in alpine coniferous forest ecosystems.

## 1. Introduction

Understory vegetation plays a critical role in maintaining forest ecosystems structure and function [1–4], facilitating energy flow and nutrient cycling and affecting canopy succession as a forest ecosystem driver [5–9]. Although the understory contributes relatively little to the total forest plant biomass [6, 7], it accounts for the largest proportion of floristic diversity [10–12]. Moreover, diverse understory vegetation increases forest structural complexity and provides habitats and food for other biotic groups, increasing their diversity [11, 13]. Understory vegetation is also particularly important to forest regeneration [4], as it can affect the germination, survival, and growth of tree seedlings by competing with them for light, water, and nutrients [1, 5, 6] or by allelopathic effects [6, 14]. Therefore, increasing attention is being paid to forest understory vegetation [15]. Understanding the factors influencing its distribution is essential for biological conservation and forest management [2, 12, 16–18].

Numerous studies have demonstrated that the species composition and diversity of understory flora can be influenced by canopy species and structure [18–21], stand management [16], ground disturbances [22, 23], light resources [24–26], litter properties [18, 27, 28], and soil nutrients and pH [3, 17, 24]. Topography can also significantly alter microclimates and resource availability under the tree canopy [19, 24, 29, 30] and in turn influence understory species composition and diversity [2, 31]. Understory vegetation in coniferous forests, hardwood forests, and mixed-wood forests has been well studied [17–19, 21, 30], and the latter two forest types are widely accepted to be more favorable to biodiversity than coniferous forests [16]. However, few studies have compared understory vegetation among coniferous species [16, 32]. In pure conifer stands, resource conditions are more homogeneous than in mixed stands, and resource quantity may be an important driver of understory species diversity [12].

Natural forest patches that are dominated by* Picea crassifolia *Kom. and* Sabina przewalskii* Kom. are widely distributed in the Qilian Mountains, northwest China. These forests are important for water conservation and preventing soil erosion in this region [33]. Typically, these two evergreen conifers form pure forests in different habitats. In this study, we investigated understory flora and associated topographic variables and site conditions in 27 plots representing these two forest types. We hypothesized that understory species composition would differ significantly between them and that juniper forest would have a more diversified understory plant community than spruce forest, because* Picea* species generally support fewer understory species than* Pinus* and* Larix* (as reviewed by Barbier et al. [16]). Additionally, we tried to determine the extent to which topographic variables and site conditions could explain the variation in understory species composition of coniferous forests.

## 2. Materials and Methods

### 2.1. Study Site

The study was carried out in the middle of the Qilian Mountains, northwest China (latitude, 38°04'–38°33'N, longitude 99°45'–100°18'E). This region has a cool-semiarid climate [34], characterized by long cold winters, short cool summers, and highly unevenly distributed precipitation. Mean annual precipitation is 447 mm, more than 80% of which occurs from May to September. Mean annual temperature is 0.6°C. The dominant tree species are* P. crassifolia* and* S*.* przewalskii*, which grow widely in northwest China [33].* S. przewalskii* is a true drought-tolerant species and prefers sunny conditions at higher elevations (2500–3500 m). In contrast,* P. crassifolia* is hygrophilous and shade-tolerant and prefers moist conditions on shaded slopes at elevations of 2300–3350 m [33]. The soil type under the tree canopy is mainly gray-brown forest soil.

### 2.2. Field Investigations

We established 27 plots of 20 × 20 m for vegetation survey at elevations ranging from 2660 m to 3480 m; 16 plots were in spruce forest and 11 plots in juniper forest. Within each plot, trees > 5.0 cm diameter at breast height (DBH) were individually surveyed for DBH and height. Total tree basal area per plot was calculated. We defined understory as shrubs and herbaceous plants growing on the forest floor. Each 20 × 20 m plot was subdivided into four 10 × 10 m quadrats, three of which were randomly selected to survey shrub species. Herbaceous species were investigated within five 1 × 1 m quadrats, one in the center and four at the corners of the 20 × 20 m plot. The height and number of individuals of each shrub and herbaceous species were measured within their respective quadrats. Percent cover of trees and herbs was visually estimated [19, 35]. Nomenclature followed* Flora Reipublicae Popularis Sinicae* (FRPS, 2004).

Elevation, aspect, slope, and slope position of each plot were recorded using a GPS and a compass meter. The aspect measurements were classified from 1 to 8 as follows: 1 (247.5°–292.5°), 2 (292.5–337.5), 3 (202.5°–247.5°), 4 (337.5–22.5), 5 (167.5°–202.5°), 6 (22.6°–67.5°), 7 (112.5°–167.5°), and 8 (67.5°–112.5°). These values are relative to east. The greater the value was, the sunnier was the site [36]. Slope position was also converted to numerical values for upper- (1), mid- (2), and down- (3) slope.

Five topsoil samples (0–10 cm depth) were randomly collected in each plot with a stainless steel cylindrical soil sampler of 5 cm in diameter. Then, we thoroughly mixed the samples in each plot to form a composite sample for subsequent analysis. Prior to analysis, the composite soil samples were air-dried and sieved to 0.2 mm for soil organic carbon (SOC) and total nitrogen (TN) analyses and to 2 mm for soil pH analysis. SOC was analyzed following the modified Mebius method [37]. TN was measured with the Kjeldahl method [38]. Soil pH was measured in a 1 : 2.5 soil to water suspension [39]. Soil bulk density was determined by using the volumetric ring method (Soil Science Society of China, 1983).

### 2.3. Data Analysis

The relative important value (IV) of each species in the understory plant community was calculated as follows:

(1) $$\begin{array}{c} \text{I}{\text{V}}_{\text{shrubs}}=\frac{\left(R_{h}+R_{a}+R_{d}\right)}{3}\\ \text{IV}{}_{\text{herbs}}=\frac{\left(R_{h}+R_{a}+R_{c}\right)}{3}, \end{array}$$

where *R*_*h*_ is relative height, defined as a species' average height as a percentage of the sum of average heights of all species; *R*_*c*_ is relative coverage, defined as a species' average coverage as a percentage of the sum of average coverage of all species; *R*_*a*_ is relative abundance, defined as the total number of individuals of a species as a percentage of the total number of individuals of all species; and *R*_*d*_ is relative dominance, the sum of a species' basal area as a percentage of total basal area of all species.

We used species richness and *α*-diversity (Shannon index, *H*′) to describe plot diversity and *β*-diversity for changes in community structure across sites within contrasting forest types [40]. *β*-diversity was calculated as follows:

(2) $$\begin{array}{c} \beta =\frac{S}{a}, \end{array}$$

where *S* is the species number in each forest type and *a* is species richness per plot. Differences in species richness and diversity of the shrub and herb layers between the forest types were tested using one-way analysis of variance with Tukey's honestly significant difference test.

Differences in understory species composition between the forest types were tested by multi-response permutation procedures (MRPP) with the Bray-Curtis index. MRPP is a nonparametric, multivariate method that provides an agreement statistic (*A*) describing the degree of within-group homogeneity compared with random expectation. In community ecology, *A*-values are generally below 0.1 and *A* > 0.3 is considered high [41]. Indicator species analysis (ISA; Dufrêne and Legendre [42]), which combines information on abundance and frequency of a species in a particular group, was used to detect species with an affinity to a certain forest type [35]. Species that were significant at the 0.05 level were considered indicator species [42]. MRPP and ISA analyses were performed with R software (R Development Core Team, 2012).

Understory species distribution considering topographic variables and site conditions was determined using the ordination method. Prior to ordination analysis, detrended correspondence analysis (DCA) was performed to select the ordination model. Since the longest DCA axis had a gradient length equal to 3.1 standard-deviation units, the unimodal model (CCA) was used to explore the relationships between understory vegetation and explanatory variables [43]. We extracted a soil proxy variable (SOIL) based on all measured soil-related variables by principal component analysis [44] and used it in the CCA ordination to avoid multicollinearity, as correlations among these variables are high (Table 1). When the variance inflation factor of selected variables was less than 10, there was no redundancy in variables [45]. Forward selection was implemented to test for significance of variables included in the model and to rank the relative importance of the individual explanatory variables [43]. Furthermore, partial canonical correspondence analysis (pCCA; ter Braak [46]) was used to partition the variation in understory species composition on topographic variables and site conditions.

## 3. Results

### 3.1. Understory Species Composition

There were significant differences in understory species composition between the two coniferous forests (observed *δ* = 0.616; expected *δ* = 0.673; *A* = 0.09; *P* < 0.001) based on MRPP analysis. Across all plots, we found 36 plant species in the forest understory; four were unique to spruce forest, and 14 occurred exclusively in juniper forest.

The ISA suggested that nine plant species were significantly associated with a particular forest type (Table 2). The majority of indicator species, including one shrub and seven herbaceous species, occurred in juniper forest, while only one species was indicative of spruce forest (Table 2).

### 3.2. Effects of Topographic Variables and Site Conditions on Understory Species Composition

In the CCA ordination, a Monte Carlo permutation test indicated that the eigenvalues for the first axis and those for all canonical axes were significant (*P* < 0.01), revealing that understory species composition was related to the measured variables (Figure 1). The first four axes explained 35.9% of the cumulative variance in species data and 83.3% of the variance in the relationship between understory species composition and environmental variables. CCA results showed that the first axis was significantly associated with elevation (*r* = −0.775), aspect (*r* = −0.474), slope (*r* = −0.464), canopy cover (*r* = 0.574), basal area (*r* = 0.467), and tree density (*r* = 0.607). The second axis was closely correlated with aspect (*r* = 0.611), slope position (*r* = 0.378), and SOIL (*r* = −0.588) (Figure 1; Table 3). Forward selection in the CCA ordination showed that understory species composition was primarily affected by elevation and aspect (*P* < 0.05; Table 4).

The pure and overlapping effects of topographic variables and site conditions were calculated by the variation partitioning model and are shown in Figure 2. The topographic variables and site conditions jointly explained 18.1% of the variation in understory species composition, of which 9.5% and 3.2% were explained by pure topographic variables and pure site conditions, respectively. Overlapping effect between topographic variables and site conditions was 5.4%. The residual fraction that remained unexplained reached up to 81.9%.

### 3.3. Understory Species Richness and Diversity

Significant differences (*P* < 0.05; Figure 3(b)) in species richness and diversity in the herb layer of the understory plant community were detected between the two forest types. Spruce forest had higher *β*-diversity and lower species richness and *α*-diversity than juniper forest (Figure 3(b)). However, there were no significant differences in species richness and diversity in the shrub layer between spruce and juniper forests (*P* > 0.05; Figure 3(a)).

## 4. Discussion

This study demonstrated a clear difference in understory species composition between plots dominated by* P*.* crassifolia *and those dominated by* S*.* przewalskii*, suggesting that changes in understory flora are related to canopy species. Understory vegetation is thought to be an ecological indicator of forest site characteristics [3, 35, 47]. Fewer understory indicator species in spruce forest imply that conditions under the spruce canopy are unfavorable for many plant species. Understory species in juniper forest were more heliophilous than those in spruce forest and included indicator species such as* Potentilla parvifolia* Fisch. ap. Lehm.,* Agropyron cristatum* (L.) Gaertn.,* Anemone cathayensis* Kitag., and* Elymus nutans* Griseb. (Table 2). The generalist species,* Carex kansuensis* Nelmes, occurred at a wide range of sites and could dominate the herb layer for several years in shaded stands [48]. It became locally abundant, making it an indicator species [49] in spruce forest.

Typically, these two forests have different distributions: juniper forest usually occurs on south-facing slopes at higher elevations, while spruce forest is found on north-facing slopes at lower elevations. In the northern hemisphere, south-facing slopes generally experience higher temperatures, greater light intensity, and lower moisture than north-facing slopes [31, 50, 51]. Understory plant species with different tolerance levels to these factors might determine their preference for a particular forest type. Because some plant species occurred exclusively in a particular forest type, the loss of that forest could result in the loss of some understory species [8, 21].

Forward selection in the CCA ordination showed that understory species distributions were strongly affected by elevation and aspect, concurring with the findings of several previous studies [2, 29, 51]. This study demonstrated a strong topographic control over understory vegetation. The SOIL variable, based on SOC, TN, soil pH, and bulk density, did not appear to strongly affect understory plant community in our study. This result contrasted with those of Qian et al. [52] and Augusto et al. [1], who reported that soil characteristics were more important than canopy species in determining understory vegetation. In addition to SOIL, other site conditions, such as canopy cover, basal area, and tree density, were not significantly related to understory species distributions.

We assessed the relative effects of topographic variables and site conditions on understory species composition and found that topographic variables were more important. This result was consistent with that obtained from CCA ordination. The proportion of variation in understory species composition that was unexplained by either topographic variables or site conditions was up to 81.9% in our study. Chávez and Macdonald [17] indicated that only 16.5% of the variation in understory species composition could be explained. A large amount of unexplained variation is a common finding [53]. The relatively low explanatory power suggests that a wide variety of unmeasured biotic and abiotic factors, dispersal strategies, stochastic events, and neighborhood effects [21, 54, 55] could exert important influences on the distributions of understory vegetation.

We found that understory species richness and diversity in the herb layers of coniferous forests varied significantly with canopy dominants. Juniper forest had higher herbaceous species richness and *α*-diversity but lower variability (*β*-diversity) across sites than spruce forest. This result points to the importance of juniper forest in maintaining biodiversity and stability in understory herbaceous communities in coniferous forests of this region. The shrub layer, however, did not differ in species richness and diversity between the two coniferous forests, suggesting that canopy species had almost no effect on understory shrubs. Light is commonly regarded as the major limiting factor affecting understory plant establishment and growth [25, 48, 56]. Generally, shade-tolerant species experience greater canopy cover and lower light transmission than shade-intolerant species [5, 57]. In this study, however, we did not find a significant difference (*P* > 0.05) in canopy cover between the two forest types. Higher species richness and *α*-diversity of the herb layer in juniper forest could partly be attributed to greater solar radiation on the south-facing slopes, which are more favorable for herbaceous species [51]. The negative correlation of understory species richness with stand basal area (*r* = −0.444, *P* < 0.05) demonstrated that understory herbs are limited by light availability [2], because higher stand basal area decreases understory light availability [58].

Several researchers have suggested that the effect of canopy species on understory species diversity may result from differences in litter thickness [1, 59]. Although litter depth was not investigated in this study, previous researches showed that spruce forest had a thicker litter layer than juniper forest [60, 61]. Augusto et al. [1] indicated that coniferous stands with thicker litter layers and shadier conditions have lower species richness, since a thick litter layer inhibits the germination and regeneration of certain herbaceous species [27, 30, 35]. To some extent, these factors explained why fewer understory species occurred in spruce forest than in juniper forest. Moreover, spruce forest is the climax plant community in this region [62]. According to the resource-ratio hypothesis [63], late successional communities will have high dominance of a few well-adapted species (e.g.,* C*.* kansuensis*) and therefore lower species richness.

Resource conditions, such as ground light and soil nutrients, may be more homogeneous in pure stands of coniferous forests because of their lower spatial and temporal variation [12, 21]. The microclimate under the spruce canopy was cool and moist [1]. Low soil temperature with a high soil C/N ratio (18.29 ± 1.11 in spruce forest; 13.86 ± 1.35 in juniper forest; *P* < 0.05) resulted in slow decomposition of organic matter [19, 24, 64]. As a result, soil available nutrients and light resources are low over the long term in spruce forest. Thus, species richness and *α*-diversity of the herb layer under the spruce canopy may not be strongly affected by interspecific competition [8, 18, 65] but rather by the poor understory conditions [1, 18, 33]. Higher light levels and lower soil C/N ratio in juniper forest together with higher herbaceous species richness suggested that resource supply controls species diversity. These results support the resource quantity hypothesis [12], which states that resource quantity is an important driver of understory species diversity at the plot scale where canopy composition is relatively uniform.

## 5. Conclusions

Understory vegetation holds a large proportion of plant diversity and contributes significantly to ecosystem functioning in forests. In this study, we compared understory vegetation in pure stands of spruce and juniper forests. Our results revealed that each forest type supported a distinct understory plant community. Forward selection showed that understory species composition was primarily affected by elevation and aspect. Comparing explanatory variables, topographic variables had higher explanatory power than did site conditions for understory species distributions based on the variation partitioning model. There was a decline in both species richness and *α*-diversity and an increase in *β*-diversity of the herb layer in the understory plant community when the canopy species shifted from* S*.* przewalskii* to* P*.* crassifolia*, highlighting the importance of the juniper forest in maintaining understory species diversity and community stability in coniferous forests. Our results improved understanding of understory species distributions in pure conifer stands.

## Figures and Tables

**Figure 1:** The CCA ordination of 27 plots and environmental variables. Arrows indicate the environmental variables (Ele, elevation; Asp, aspect; Slo, slope; Pos, slope position; BA, basal area; Cov, canopy cover; Den, tree density). Plots dominated by* P*.* crassifolia *and* S*.* przewalskii *are represented by circles (*n* = 16) and squares (*n* = 11), respectively.

**Figure 2:** Partition the variation in understory species composition on topographic variables and site conditions. Pure and overlapping effects: (a) pure topography; (b) pure site conditions; (c) overlapping effects; (d) residual.

**Figure 3:** Comparison of species richness, *α*- and *β*-diversity of the shrub and herb layers of understory plant community between spruce and juniper forests.

**Table 1:** Correlation analysis of soil-related variables (*n* = 27).

	SOC	TN	pH
TN	0.933∗∗		
pH	−0.843∗∗	−0.861∗∗	
BD	−0.799∗∗	−0.749∗∗	0.631∗∗

SOC: soil organic carbon; TN: total nitrogen; BD: soil bulk density.

**P < 0.01.

**Table 2:** Species identified as significant indicators of spruce or juniper coniferous forests, based on indicator species analysis.

Forest type	Indicator species	Indicator value	*P*
Spruce forest	*Carex kansuensis* Nelmes	0.648	0.013

Juniper forest	*Potentilla parvifolia* Fisch. ap. Lehm.	0.709	0.003
	*Kobresia myosuroides* (Villars) Fiori	0.545	0.002
	*Potentilla saundersiana* Royle	0.364	0.023
	*Saussurea japonica* (Thunb.) DC.	0.273	0.047
	*Agropyron cristatum* (L.) Gaertn.	0.505	0.002
	*Anemone cathayensis* Kitag.	0.364	0.023
	*Ranunculus tanguticus* (Maxim.) Ovcz.	0.636	0.001
	*Elymus nutans* Griseb.	0.364	0.019

**Table 3:** Results of the CCA showed correlation coefficients between environmental variables and the CCA axes, species-environment correlation, cumulative variance relationship with the four axes, and variance inflation factor of each environmental variable (VIF).

Variables	Axis 1	Axis 2	Axis 3	Axis 4	VIF
Elevation	−0.775∗∗∗	−0.302	−0.149	0.089	2.52
Aspect	−0.474∗	0.611∗∗∗	−0.110	0.087	1.83
Slope position	0.318	0.378∗	−0.132	−0.273	1.79
Slope	−0.464∗	−0.089	−0.132	−0.311	1.65
SOIL	−0.159	−0.588∗∗	−0.069	0.304	1.72
Canopy cover	0.574∗∗	−0.079	−0.006	0.066	2.49
Basal area	0.467∗	−0.066	−0.346	−0.050	1.97
Tree density	0.607∗∗∗	−0.083	0.303	−0.238	3.25
Species-environment correlations	0.907	0.908	0.840	0.713	
Cumulative percentage variance					
Of species data	13.9	25.1	32.1	35.9	
Of species-environment relation	32.3	58.3	74.5	83.3	

*P < 0.05; **P < 0.01; ***P < 0.001.

**Table 4:** Marginal and conditional effects of each environmental variable obtained from the forward selection in the CCA ordination.

Variables	Marginal effect	Conditional effect	*F*	*P*
	*λ*_1_	*λ*_*A*_		
Elevation	0.36	0.36	3.37	0.002∗∗
Aspect	0.29	0.28	2.77	0.002∗∗
Slope position	0.16	0.10	1.09	0.370
Slope	0.17	0.10	1.03	0.404
SOIL	0.19	0.09	0.95	0.534
Canopy cover	0.20	0.08	0.75	0.726
Basal area	0.18	0.16	1.66	0.058
Tree density	0.25	0.14	1.53	0.056

**P < 0.01.
